RETRACTED

# The efficiency and safety of tranexamic acid for reducing blood loss in open myomectomy: A meta-analysis of randomized controlled trials

**DOI:** 10.1097/MD.0000000000007072

**Published:** 2017-06-08

**Authors:** Dongdong Wang, Lixia Wang, Yifei Wang, Xinyan Lin

**Affiliations:** a Department of Neurology; b Department of Gynaecology and Obstetrics, The Second Hospital of Dalian Medical University, Liaoning, China.

**Keywords:** blood loss, blood transfusion, meta-analysis, open myomectomy, tranexamic acid

## Abstract

**Objective:**

This meta-analysis aimed to perform a meta-analysis including randomized controlled trials (RCTs) to assess the efficiency and safety of tranexamic acid (TXA) for reducing blood loss and transfusion requirements in patients undergoing open myomectomy.

**Methods:**

A systematic search was performed in Medline (1966–2017.03), PubMed (1966–2017.03), Embase (1980–2017.03), ScienceDirect (1985–2017.03,) and the Cochrane Library. Study evaluated the efficiency and safety of TXA in myomectomy was selected. Meta-analysis was performed using Stata 11.0 software.

**Results:**

Four RCTs including 328 patients met the inclusion criteria. The present meta-analysis indicated that there were significant differences between groups in terms of total blood loss (standard mean difference [SMD] = −1.512, 95% confidence interval [CI]: −2.746 to −0.278, *P* = .016), postoperative hemoglobin level (SMD = 0.650, 95% CI: 0.045–1.255, *P* = .035), transfusion requirements (SMD = −0.102, 95% CI: −0.199 to −0.006, *P* = .038), and duration of surgery (SMD = −0.514, 95% CI: −0.749 to −0.280, *P* = .000). In addition, no adverse effect was identified in treatment groups.

**Conclusions:**

Intravenous administration of TXA in open myomectomy was associated with significantly reduced total blood loss, postoperative hemoglobin decline, duration of surgery, and transfusion requirements. Based on the limitations of the current meta-analysis, high-quality RCTs with long-term follow-up are still required.

## 1 Introduction

Uterine fibroids are common benign gynecologic tumors and 25% to 30% of women would be diagnosed at a time during their lives.^[1]^ It could be located at different sites and sometimes implants the uterine cavity. The common symptoms are bellyache, leukorrhagia, menorrhagia, and symptomatic anemia. More importantly, uterine fibroids have a potential impact on fertility. Previous studies have reported that infertility was related to submucosal fibroids^[2]^; however, it is unclear with regards to the effect of intramural fibroids.

Various methods are available for the treatment of symptomatic myomas including medical and surgical intervention.^[3,4]^ Myomectomy remains the most popular methods for those who have myomas and desire further childbearing. However, substantial perioperative blood loss has been associated with surgical procedure and sometimes hysterectomy has to be performed to control bleeding which results in increased morbidity and mortality. Many strategies have been used to manage blood loss including mechanical tourniquets, administration of hemostatic agents, autologous donation and minimally invasive procedures.^[5–7]^ However, blood transfusions were still required to treat anemia in many cases. Allogenic blood transfusion would increase the risk of adverse events, such as virus infections, immunologically mediated diseases, and cardiovascular dysfunction, resulting in a financial burden and potentially life-threatening effects on patients.^[8,9]^

Recently, the use of tranexamic acid (TXA) has become popularized in surgical procedure. TXA is a synthetic analog of an amino acid whose biological activity inhibits plasminogen from dissolving clots.^[10]^ In previous studies, the administration of TXA was reported to be associated with reduced perioperative blood loss and transfusion units in cardiac surgery, orthopedic surgery, and organ transplantation.^[11–13]^

Currently, the application of TXA in myomectomy was seldom reported. Thus, there is a lack of scientific evidence regarding the hemostatic effect of TXA in myomectomy. Therefore, we perform a meta-analysis of randomized controlled trials (RCTs) to assess the efficiency and safety of TXA for reducing blood loss and transfusion requirements in patients undergoing myomectomy.

RETRACTED

## 2 Methods

### 2.1 Search strategy

Electronic databases were systemically searched including Embase (1980–2017.03), Medline (1966–2017.03), PubMed (1966–2017.03), ScienceDirect (1985–2017.03), web of science (1950–2017.03), and Cochrane Library for potential relevant studies. Reference lists of all the potential included studies and relevant reviews were hand-searched for any additional trials. No restrictions were imposed on language. The search terms “Tranexamic acid”, “myomectomy’,’ and “blood loss” were used in combination with Boolean operators AND or OR. The retrieval process is presented in Figure 1. The study was approved by the ethics committee of the Second Hospital of Dalian Medical University.

**Figure 1:** Search results and the selection procedure.

### 2.2 Inclusion and exclusion criteria

Studies were considered eligible if they met the following criteria: published clinical RCTs; patients undergoing open myomectomy experiment group received intravenous TXA for blood management and control group received placebo or nothing; the primary outcomes included total blood loss, postoperative hemoglobin level, transfusion rate, and drainage volume. Secondary outcomes included duration of surgery and postoperative adverse effects such as deep vein thrombosis (DVT) and pulmonary embolism (PE). Studies would be excluded from current meta-analysis for incomplete data, case reports, conference abstract, or review articles.

RETRACTED

### 2.3 Selection criteria

Two authors independently reviewed all the abstracts of the potential studies identified by the above searches. After an initial decision, full text of the studies that potentially met the inclusion criteria was reviewed and final decision was made. A senior reviewer is consulted in case of disagreement regarding which studies to include.

### 2.4 Date extraction

A standard form for date extraction is printed for date extraction. Two authors independently extracted the relevant data from the included articles. Details of incomplete data of included studies are obtained by consulting the corresponding author. Following data were extracted: first author names, published year, sample size, study design, comparable baseline, dosage of TXA, and duration of follow-up. Other relevant data were also extracted from individual studies.

### 2.5 Quality assessment

Quality assessment of the included studies was assessed by 2 authors independently. Modified Jadad score (7-point scale), which was based on Cochrane Handbook for Systematic Reviews of Interventions, is used for assessment of RCTs. Studies which score >4 points were considered high-quality. We conducted “risk of bias” table including the following key points: random sequence generation, allocation concealment, blinding, incomplete outcome data, free of selective reporting, and other bias; each item was recorded by “Yes,” “No,” or “Unclear.”

The qualities of evidence of main outcomes in present meta-analysis were evaluated using the Recommendations Assessment, Development, and Evaluation (GRADE) system including the following items: risk of bias, inconsistency, indirectness, imprecision, and publication bias. The recommendation level of evidence is classified into the following categories: high, which means that further research is unlikely to change confidence in the effect estimate; moderate, which means that further research is likely to significantly change confidence in the effect estimate and may change the estimate; low, which means that further research is likely to significantly change confidence in the effect estimate and to change the estimate; very low, which means that any effect estimate is uncertain.

### 2.6 Data analysis and statistical methods

All calculations were performed using Stata 11.0 software (The Cochrane Collaboration, Oxford, United Kingdom). Statistical heterogeneity was assessed based on the value of *P* and *I*^2^ using standard *χ*^2^ test. When *I*^2^ >50%, and *P* < .1 was considered to be of significant heterogeneity, random-effect model was performed for meta-analysis. Otherwise, fixed-effect model was used. If possible, sensibility analysis is conducted to explore the origins of heterogeneity. The results of dichotomous outcomes were expressed as risk difference (RD) with 95% confidence intervals (CIs). For continuous various outcomes, mean difference and standard mean difference (SMD) with a 95% CI was applied for assessment. Sensitivity analysis was conducted for the main results according to the dosage of TXA.

RETRACTED

## 3 Results

### 3.1 Search result

A total of 458 studies were preliminarily reviewed. By screening the titles and reading the abstracts and entire contents, 454 reports were excluded from present meta-analysis following inclusion criteria. No gray reference was included. Finally, 4 RCTs,^[14–17]^ which had been published between 2008 and 2016, were enrolled in the present meta-analysis and include 164 patients in the TXA groups and 164 patients in the control groups.

### 3.2 Study characteristics

Demographic characteristics, the details about the included studies are summarized in Table 1. The sample size of the included studies ranged from 34 to 132. All of them evaluated the efficiency and safety of TXA for reducing blood loss in open myomectomy. Experimental groups received intravenous TXA, whereas control groups received placebo or none. There is a variation in dosage of TXA in experimental groups. Three studies^[14,16,17]^ performed general anesthesia and 1^[15]^ did not give a detailed description. All ^[14–17]^ studies reported that open myomectomy was performed by same team. The indication of blood transfusion was based on postoperative hemoglobin level. None of the included studies performed a sample size calculation. All of them suggest the outcomes for at least 95% of the patients. The follow-up period ranged from 1 to 2 months.

**Table 1:** Cohort characteristics.

### 3.3 Risk of bias assessment

Modified Jadad score, which was based on Cochrane Handbook for Systematic Reviews of Interventions, is used for assessment of RCTs (Table 2). All of the RCTs reported a clear inclusion and exclusion criteria and suggest a methodology of randomization; all of them demonstrated that randomization sequence was generated by computer. Three of them^[14–16]^ reported allocate concealment was achieved by sealed envelopes. Double blinding was provided in 3 RCTs.^[15–17]^ Only one^[15]^ of them had attempted to blind assessors. Each risk of bias item is presented as the percentage across all included studies, which indicates the proportion of different levels of risk of bias for each item (Table 3). All RCTs provided complete outcome data. None of them performed intent-to-treatment analysis; thus, a potential risk for type II statistical error would exist.

RETRACTED

**Table 2:** Methodological quality of the randomized controlled trials.

**Table 3:** Risk of bias.

### 3.4 Outcomes for meta-analysis

#### 3.4.1 Total blood loss

Four studies^[14–17]^ reported total blood loss following open myomectomy. Statistical heterogeneity was observed in present meta-analysis (*χ*^2^ = 65.74, df = 3, *I*^2^ = 95.4%, *P* = .000); therefore, a random-effects model was applied. We found that there was significant difference between the TXA groups and control groups regarding the total blood loss (SMD = −1.512, 95% CI: −2.746 to −0.278, *P* = .016; Fig. 2).

**Figure 2:** Forest plot diagram showing effect of intravenous tranexamic acid on total blood loss.

#### 3.4.2 Postoperative hemoglobin level

Four studies^[14–17]^ reported postoperative hemoglobin level following open myomectomy. There was significant heterogeneity (*χ*^2^ = 19.45, df = 3, *I*^2^ = 84.6%, *P* = .000); therefore, a random-effects model was used. The result of meta-analysis showed that there was significant difference between the TXA groups and control groups regarding the postoperative hemoglobin level (SMD = 0.650, 95% CI: 0.045–1.255, *P* = .035; Fig. 3).

**Figure 3:** Forest plot diagram showing effect of intravenous tranexamic acid on postoperative hemoglobin level.

#### 3.4.3 Transfusion requirements

Transfusion requirements following open myomectomy were presented in 4 studies.^[14–17]^ There was no significant heterogeneity (*χ*^2^ = 4.93, df = 3, *I*^2^ = 39.2%, *P* = .177) and a fixed-effects model was used. The present meta-analysis showed that there was significant difference between the TXA and control groups in terms of transfusion requirement (SMD = −0.102, 95% CI: −0.199 to −0.006, *P* = .038; Fig. 4).

**Figure 4:** Forest plot diagram showing effect of intravenous tranexamic acid on transfusion requirements.

#### 3.4.4 During of surgery

Three studies^[14,16,17]^ provided the operation time among studies. No significant heterogeneity was found (*χ*^2^ = 4.73, df = 2, *I*^2^ = 57.8%, *P* = .094); therefore, a fixed-effects model was used. Meta-analysis revealed that there was significant difference between the TXA and control groups in terms of duration of surgery (SMD = −0.514, 95% CI: −0.749 to −0.280, *P* = .000; Fig. 5).

**Figure 5:** Forest plot diagram showing effect of intravenous tranexamic acid on duration of surgery.

RETRACTED

#### 3.4.5 DVT

Four articles^[14–17]^ reported the incidence of DVT following open myomectomy. A fixed-effects model was used because of the low significant heterogeneity among these studies (*χ*^2^ = 0.50, df = 3, *I*^2^ = 0%, *P* = .919). No significant difference was found between the groups (RD = 0.000, 95% CI: −0.036 to 0.036, *P* = .999; Fig. 6).

**Figure 6:** Forest plot diagram showing effect of intravenous tranexamic acid on risk of deep vein thrombosis.

#### 3.4.6 PE

PE was reported in 4 studies.^[14–17]^ A fixed-effects model was used because no significant heterogeneity was found among the studies (*χ*^2^ = 0.66, df = 2, *I*^2^ = 0%, *P* = .717). No significant difference was found in the PE incidence between the 2 groups (RD = 0.007, 95% CI: −0.020 to 0.033, *P* = .617; Fig. 7).

**Figure 7:** Forest plot diagram showing effect of intravenous tranexamic acid on risk of pulmonary embolism.

#### 3.4.7 Sensitivity analysis

Sensitivity analysis was conducted for the main results according to the dosage of TXA, which is presented in Table 4.

**Table 4:** The outcome of sensitivity analysis for main results.

## 4 Discussion

To the best of our knowledge, this study is the first meta-analysis from RCTs to assess the efficiency and safety of TXA for reducing blood loss and transfusion requirements in patients undergoing myomectomy. The most important finding of the present meta-analysis was that the intravenous application of TXA could significantly reduce the total blood loss, hemoglobin decline, and transfusion requirements after open myomectomy. Moreover, no increased risk of the incidence of DVT and or PE was identified. All outcomes in this meta-analysis were evaluated using the GRADE system. The evidence quality for each outcome was high to moderate (Table 5), which means that further research is likely to significantly change confidence in the effect estimate and may change the estimate.

**Table 5:** The GRADE evidence quality for main outcome.

TXA, which acts as antifibrinolytic agent, is famous for proven success in reducing peri- and postoperative blood loss and widely used in surgical procedure. Konig et al^[18]^ reported that topical application of TXA for patients undergoing primary total hip arthroplasty is effective and safe. Fu et al^[19]^ conducted a meta-analysis from 22 RCTs and showed that TXA is beneficial for patients undergoing total knee arthroplasty, which can significantly reduce total blood loss. Recently, TXA has been studied in gynecology and obstetrics field. Previous articles have reported that TXA acts as a nonhormonal treatment for excessive hemorrhage during the menstrual period.^[20]^

Uterine fibroid represents a major health issue with an estimated 234 million women affected all over the world. Symptomatic fibroid that required intervention accounts for about 25% of all cases.^[21]^ Myomectomy is one of the most common surgical procedures for treatment of the uterine fibroid, which may be associated with massive perioperative blood loss. With the advanced of surgical techniques, there was a significantly reduced hemorrhage during operation. Laparoscopic myomectomy is an alternative to the abdominal approach with fewer complications and shortened hospital stay.^[22]^ Although it has been proved to be beneficial on blood management, the surgical indication depends on the size, number, and location of the myoma, which limited the clinical application. Therefore, open myomectomy is widely performed; however, it was associated with more hemorrhage from tissue and vessels dissection that might necessitate hysterectomy resulting in increased morbidity and mortality.

RETRACTED

TXA can be applied by various routes including intravenous, oral, and intramuscular. The optimal routes of TXA have been more studied in orthopedic and cardiac surgery. All included patients received intravenous TXA and the dose of TXA differed between trials. TXA can inhibit the activation of plasminogen by plasminogen activator and blocks the lysine-binding sites of plasminogen to fibrin.^[23]^ Previous fundamental research has reported that the levels of plasminogen activators increased 30 minutes after the initiation of surgery.^[24]^ Thus, the theoretical basis could explain a potential efficiency for reducing blood loss for surgical procedures. The present meta-analysis indicated that intravenous TXA could significantly decrease total blood loss and hemoglobin decline following open myomectomy. Significant heterogeneity was identified regarding the target parameters and it would be influenced by several factors such as anesthesia methods, dosage of TXA, and surgical technique. Considering that only 4 RCTs were included in present meta-analysis, we did not perform a subgroup analysis. More high-quality RCTs are necessary in subsequent research.

Although effective strategies have attempted for reducing blood loss, allogeneic blood transfusions were still required for treatment anemia. However, blood transfusion would be associated with potential adverse effects, for instance, infections disorder, hemolytic reaction, and anaphylactic reaction among others. Currently, whether intravenous TXA could decrease transfusion requirements in open myomectomy remains controversial. Shaaban et al^[14]^ showed that the transfusion rate was significantly reduced when applied intravenous TXA (*P* < .01). However, Caglar et al^[16]^ reported similar blood transfusion requirements between treatment groups (*P* = .25). Meta-analysis is performed as major statistical method in the present study. It could strengthen statistical power and enlarge sample size by pooling results of published articles that could point out stronger evidence. In addition, no guidelines have been proposed to normalize the administration of TXA in open myomectomy. Thus, there is a requirement for an evidence base to help gynecologists make clinical decisions. The present meta-analysis indicated that the intravenous application of TXA was associated with a further significant reduction in the transfusion requirements. Another important finding of the present meta-analysis was that intravenous TXA could significantly shorten the duration of surgery. The result may explain that intraoperative blood loss would be decreased and there is less time for hemostasis process. Moreover, lower transfusion rate also spent less time.

RETRACTED

DVT has been identified as a common complication that may develop into PE and even result in death following surgery.^[25]^ Previous studies have reported a higher risk of DVT and PE when they utilized TXA. This finding may be because of its antifibrinolytic effect. The present meta-analysis indicated that there was no significant difference regarding the incidence of DVT or PE. Although the methods of thromboprophylaxis differed among included studies, no significant heterogeneity was showed in pooled results. However, owing to the limitation of the included studies, larger sample size with longer follow-up is required to confirm whether the intravenous TXA is safe without increasing thrombotic events.

Several potential limitations of this study should be noted. First, only 4 RCTs were included, and the sample size was relatively small. Second, some important outcome parameters such as drainage volume and range of motion were not fully described and could not be included in the meta-analysis. Third, because of the limited number of included studies, subgroup analyses were not performed for total blood loss and postoperative hemoglobin level; therefore, we could not determine the sources of heterogeneity. Fourth, short-term follow-up may lead to the underestimation of complications. Lastly, publication bias is an inherent weakness that exists in all meta-analyses.

Despite the aforementioned limitations, this study is the first meta-analysis to pool the results from randomized controlled trials to evaluate the efficiency and safety of TXA for reducing blood loss in patients undergoing open myomectomy. High-quality RCTs with long-term follow-up are needed to explore optimal dose, appropriate application methods, and adverse effects in future studies.

RETRACTED

## 5 Conclusions

Intravenous administration of TXA in open myomectomy was associated with significantly reduced total blood loss, postoperative hemoglobin decline, duration of surgery, and transfusion requirements. Based on the limitations of the current meta-analysis, high-quality RCTs with long-term follow-up are still required.
